The article "Leukobiopsy – A Possible New Liquid Biopsy Platform for Detecting Oncogenic Mutations" was published in 2020. Journal: Front Pharmacol.

# Leukobiopsy – A Possible New Liquid Biopsy Platform for Detecting Oncogenic Mutations

**DOI:** 10.3389/fphar.2019.01608

**Published:** 2020-01-24

**Authors:** Shilpa Chennakrishnaiah, Thupten Tsering, Saro Aprikian, Janusz Rak

**Affiliations:** Montreal Children's Hospital, RI MUHC, McGill University, Montreal, QC, Canada

**Keywords:** oncogenes, neutrophils, extracellular vesicles, exosomes, thrombosis, liquid biopsy, cancer, diagnosis

## Abstract

Detection of unique oncogenic alterations encoded by the sequence or biochemical modification in cancer-associated transforming macromolecules has revolutionized diagnosis, classification and management of human cancers. While these signatures were traditionally regarded as largely intracellular and confined to the tumor mass, oncogenic mutations and actionable cancer-related molecular alterations can also be accessed remotely through their recovery from biofluids of either rare circulating tumor cells (CTCs), or of more abundant non-cellular carriers, such as extracellular vesicles (EVs), protein complexes, or cell-free tumor DNA (ctDNA). Tumor-related macromolecules may also accumulate in circulating platelets. Collectively, these approaches are known as liquid biopsy and hold promise as non-invasive, real-time opportunities to access to the evolving molecular landscape of human malignancies. More recently, a possibility of recovering cancer-specific DNA sequences from circulating leukocytes has also been postulated using experimental models. While it is often assumed that these and other liquid biopsy approaches rely on material passively shed from the tumor mass or its debris, recent evidence suggests that several regulated processes contribute to the abundance, nature, half-life, and turnover of different circulating cancer-related molecular signals. Moreover, many of these signals possess biological activity and may elicit local and systemic regulatory responses. Thus, a better understanding of the biology of liquid biopsy platforms and analytes may enable achieving improved performance of this promising and emerging diagnostic strategy in cancer.

## Introduction

In this overview we wish to articulate and contextualize two frequently overlooked considerations. First, the liquid biopsy paradigm sweeping through the diagnostic space in cancer might have an important functional component as the respective analytes, be it soluble nucleic acids or circulating cells are under influence of regulatory processes that control their abundance. They also may possess poorly understood biological activities of their own. Second, the list of biological carriers that can be remotely intercepted and used as liquid biopsy diagnosis platforms continues to expand, one novel possible addition being leukocyte cargo of cancer-related nucleic acids, that can be retrieved in the process that can be termed “leukobiopsy”. While we discuss the necessary context of these considerations this article is not intended as a systematic overview of liquid biopsy as such, a topic that has been amply covered by leaders in the field as, at least partially, reflected in citations used in the remainder of the text.

## Liquid Biopsy Platforms in Cancer

It could be argued that progress achieved in the management of human cancers during the past several decades is largely attributable to a better understanding of the biological, cellular and molecular underpinnings of different malignant states (Vogelstein and Kinzler, 2004). While functional significance of the hallmarks of cancer (Hanahan and Weinberg, 2011) has illuminated the salient commonalities of neoplastic processes, it is the understanding of tumor diversity, existence of disease subtypes, and aspects of their molecular uniqueness, that has guided successes in targeted and biological therapy efforts (Gotwals et al., 2017). Indeed, it can be argued that differences between disease entities are often more actionable than similarities.

The centrepiece in this paradigm and the source of hope for developing more effective, personalized anticancer treatment strategies, is the notion of striking at crucial oncogenic drivers, either genetic or epigenetic, that are implicated in cancer causation (Vogelstein and Kinzler, 2004), but which may be highly context-specific (Ben-David et al., 2019). While compiling the related molecular information is often illuminating, and has led to the discovery of new therapeutic targets as well as the remarkable molecular diversity of major human cancers (Curtis et al., 2012; Reifenberger et al., 2017), it does not necessarily, by itself, lead to successful therapies for several reasons. First, driver genes often unleash a chain reaction of stromal and host responses, such as angiogenesis (Rak et al., 1995), inflammation (Sparmann and Bar-Sagi, 2004), immunosuppression (Spranger and Gajewski, 2018), coagulopathy (Yu et al., 2005), or other complex microenvironmental changes (Finak et al., 2008), which assume a pathogenetic role of their own (Magnus et al., 2014) and may not be readily reversible even upon suppression of the oncogenic signal. Second, the genetic evolution of cancer cell clones generates perpetual drift in their oncogenic repertoires, resulting in heterogeneity and co-existence of several disease-causing mechanisms often obscured by dominant cell populations (Gerlinger et al., 2012; Ben-David et al., 2019). Third, processes of invasion and metastasis result in the formation of a multifocal malignant disease where different tumors progress independently in the same individual (Fidler, 2003; Gerlinger et al., 2012). Fourth, anticancer therapies often result in a profound re-alignment of the molecular repertoire of cancer cell populations, due to mutations, selection, or the entry of minor clones into the disease process (Johnson et al., 2014; Wang et al., 2016; Garnier et al., 2018). This happens at the time when the recurrent disease no longer responds to prior therapy, while new vulnerabilities are often still unknown (Wang et al., 2016).

These biological considerations complicate molecular diagnosis of cancers, which is traditionally predicated on the analysis of surgical or biopsy tissue specimens. Such one-time snapshots of limited spectrum of tumor microregions is simply insufficient to accurately reflect the spatial and temporal complexity and cellular heterogeneity of the progressive and evolving disease (Siravegna et al., 2017). While serial biopsy programs may alleviate these challenges, at least to some extent, the invasive nature of these procedures, risk of complications, tissue sampling errors, ethical considerations and inaccessibility of anatomically difficult sites or disseminated tumor foci may severely curtail the expected gains (Siravegna et al., 2017).

Many (if not all) human cancers, even if anatomically localized, exert a level of systemic impact through the release of tumor cells and their products into biofluids, such as blood, cerebrospinal fluid, urine, ascites, pleural effusion, or glandular secretions. Collection and analysis of these remote signals, long known as liquid biopsy (**Figure 1**), offers a remote, continuous and non-invasive access to salient characteristics of all tumor cell subpopulations (and stroma) with adequate representation in the appropriate biofluid (Pantel and Alix-Panabieres, 2019). While this is an area of intense interest, and one extensively reviewed in recent literature (Crowley et al., 2013; Siravegna et al., 2017; Wan et al., 2017; Heitzer et al., 2019; Pantel and Alix-Panabieres, 2019), it deserves a few general comments and context.

**Figure 1:** Liquid biopsy platforms and processes that regulate them in cancer. Several processes affect the state of biofluids (right) and their content of liquid biopsy analytes. Each form of liquid biopsy (CTCs, cfDNA, EVs, platelets, and leukocytes) may be affected by unique regulatory influences that may change the content of biological information (see text for details).

First, the nature of tumor-related material that is recovered from biofluids, such as plasma, ranges from simple molecular biomarkers such as PSA, CA125, or CEA to more comprehensive representations of cancer complexity and driving mechanisms (bona fide liquid biopsy), such as circulating tumor cells (CTCs) (Pantel and Alix-Panabieres, 2019), circulating cell-free DNA (cfDNA) (Schwarzenbach et al., 2011), tumor-educated platelets (TEPs) carrying tumor-related biomolecules (Cervi et al., 2008), especially RNA (Nilsson et al., 2011; In ‘t Veld and Wurdinger, 2019), and an array of extracellular particles (EPs) and vesicles (EVs) containing molecular and mutational fingerprints (proteins, RNA and DNA) of their donor cancer cells (Al-Nedawi et al., 2008; Skog et al., 2008; Balaj et al., 2011; Kahlert et al., 2014; Lazaro-Ibanez et al., 2014; Lee et al., 2014; Thakur et al., 2014; Siravegna et al., 2017; Miller et al., 2019). Each of these liquid biopsy platforms is based on a different, defined or presumed biological process resulting in the shedding of cancer-related material into the circulation. For example, while CTCs are generally believed to represent a part of (though not tantamount to) the metastatic intravasation process, ctDNA is often viewed as a result of cellular breakdown and release of debris from the tumor mass or from other poorly defined release mechanisms (Siravegna et al., 2017).

By their very nature, different liquid biopsy platforms pose different analytical challenges. For example, the relative abundance of CTCs is thought to be low (1–10 CTCs/ml of plasma), which underrepresents the cellular heterogeneity of the corresponding cancer, while ctDNA is often present at low levels, but more importantly, in a largely fragmented molecular form. Extraction of RNA signals from circulating ribonucleoprotein complexes, platelets or EVs may be technically complex and burdened with variability (Das et al., 2019; Jeppesen et al., 2019). While some of these challenges are often perceived as “technical” in nature, they may result from our limited understanding of the biological processes leading to the presence of specific liquid biopsy forms and analytes in biofluids, as well as mechanisms regulating the fate, half-life, content and diagnostic meaning of the related molecular signals.

## Extracellular Vesicles as Carriers of Diagnostic Information

EV/EPs exemplify the link between cancer biology and its extracellular and systemic representation (Rak, 2013). Cells are programmed to export complex multi-molecular packets either as membrane-less EPs, such as exomeres (Zhang et al., 2018), or as a wide spectrum of EVs (Zijlstra and Di Vizio, 2018), of which exosomes originate intracellularly, within the late endosome, while ectosomes (microvesicles) and many other EVs result from outward budding of the plasma membrane (Van Niel et al., 2018).

Apart from their unique biogenesis, exosomes possess several distinctive properties. They tend to be under 150 nm in size, float at low density of sucrose (1.11–1.19) and carry a repertoire of surface markers enriched in tertraspanins (CD9, CD63, CD81, and CD82), components of endosomal sorting complex required for transport (ESCRT; TSG101) and related proteins (ALIX, Syntenin 1). While this places ESCRT at the centre of EV biogenesis, exosomes may also be generated in an ESCRT-independent manner linked to production of ceramide within the vesicle membrane by neutral sphingomyelinases (SMPD3) (Van Niel et al., 2018; Xu et al., 2018). Therefore, inhibitors of SMPD3 may reduce cellular exosome production (Trajkovic et al., 2008), as could targeting elements of vesicular transport system (Rab27a/b, SYT7) or tetraspanins (Chairoungdua et al., 2010; Luga et al., 2012; Sung et al., 2015).

Budding from the plasma membrane gives rise to a large spectrum of EVs ranging from 40nm–100nm (ARMMs), 150–1,000 nm (microvesicles), over 1um (migrasomes), and 1um–10 um (large oncosomes) with different properties, biogenetic origins, cargo packaging mechanisms, molecular make ups and biological activities, as reviewed extensively in the recent literature (Muralidharan-Chari et al., 2009; Thery et al., 2009; Abels and Breakefield, 2016; Kowal et al., 2016; French et al., 2017; Xu et al., 2018; Jeppesen et al., 2019). Moreover, molecular predictions based on the composition of the EV proteome suggest the existence of even greater diversity (dozens or more) of distinct EV subtypes that are only beginning to emerge. Efforts are underway to map EV landscapes (Choi et al., 2017) in various settings using single EV analysis afforded by nano-flow cytometry (Nolan, 2015; Choi et al., 2018) and microfluidics (Fraser et al., 2019).

EVs represent a conserved regulatory mechanism spanning the evolutionary spectrum from prokaryotic (Ibanez de Aldecoa et al., 2017) to mammalian cells (Van Niel et al., 2018) and endowed with two fundamentally important functions. First, EVs enable a rapid active expulsion of large amounts of molecular material including effector and signalling proteins, as well as lipids, RNA, and DNA from their parental cells. This may enable cellular adaptation to differentiation programs (Johnstone, 2006), noxious signalling events (Chairoungdua et al., 2010), as well as molecular (Takahashi et al., 2017) and therapeutic stresses (Montermini et al., 2015; Garnier et al., 2018). Second, EVs are capable of delivering their molecular content to other cells thereby mediating intercellular communication, integration and molecular flux (Mulcahy et al., 2014). In cancer, EVs mediate transmission of mutant oncogenes between cells resulting in biological responses resembling malignant transformation (Al-Nedawi et al., 2008; Lee et al., 2016; Choi et al., 2017). Both of these properties (expulsion and uptake) are relevant for the emerging diagnostic use of EVs in cancer and other diseases.

From the liquid biopsy perspective EVs offer unprecedented advantages, but also pose some challenges. For example, in cancer, tumor-derived EVs carry a wealth of clinically important information as to driver mutations (Al-Nedawi et al., 2008; Skog et al., 2008; Choi et al., 2017), drug resistance markers (Bebawy et al., 2009; Boelens et al., 2014), determinants of immunoregulation (e.g. PD-L1) (Ricklefs et al., 2018) and other salient features of tumor and stroma. With up to 10^12^ EVs per ml of plasma, EVs exceed numbers of CTCs (<10 per ml) by several orders of magnitude, which also translates into favorable complexity profiles, which likely approximates the representation of the true heterogeneity of parental cancer cell populations. Unlike tumor-educated platelets that may undergo activation and sequestration, EVs circulate in biofluids in relatively stable biological form. Unlike ctDNA, EVs co-express informative and diverse biological signals, such as nucleic acid sequences and protein lineage markers, which makes them amenable to multiplexing and tracing cellular sources of cargo (Choi et al., 2017). This may enhance the specificity of detection and offer several other advantages (Shao et al., 2015; Zachariah et al., 2018). Moreover, EVs protect their molecular cargo from degradation and enable recovery of meaningful signals even from archival samples (Skog et al., 2008).

On the other hand, the abundance of cancer-related EVs in blood is estimated to be low, in single digit percentages (Abels and Breakefield, 2016), which poses sensitivity and background challenges. Their heterogeneous content of informative signals (Choi et al., 2019) may further impact detectability, all of which is compounded by a poor understanding of cargo packaging mechanisms, their regulation, and of the processes governing EV half-lives and fate upon entry into biofluids (Peinado et al., 2012; Hoshino et al., 2015; Chennakrishnaiah et al., 2018; Thery et al., 2018).

## Leukobiopsy

While bolus injection of EVs into the circulation leads to their rapid elimination within minutes to hours, due to the uptake in major organs (liver, spleen) (Wang et al., 2012; Thery et al., 2018), less is known about the natural turnover of EVs released into the circulation spontaneously. Notably, CD47 expression (“don't eat me signal”) prolongs the half life of exosomes in the circulation suggesting that their uptake by phagocytes controls their fate (Kamerkar et al., 2017). Such uptake can also be demonstrated directly by EV-mediated transfer of cancer-related signalling receptors (e.g. MET)(Peinado et al., 2012), or RNA (Ridder et al., 2015) from cancer cells to myeloid cells *in vivo*.

Since the half-life of circulating blood cells is much longer than that of EVs and varies between 8 h for neutrophils (Summers et al., 2010), 3 days for monocytes (Patel et al., 2017) to 120 days for red blood cells (Franco, 2012), their possible retention of EV related material could prolong the availability of such molecules in the circulation. For this reason we assessed the distribution in blood of oncogenic DNA associated with the EV fraction of the cellular secretome in the case of cancer cells driven by either mutant HRAS (Lee et al., 2014) or amplified HER2 oncogenes (Chennakrishnaiah et al., 2018). The respective cancer cell lines (RAS3 and BT474) were inoculated into immune deficient mice and once tumors were established and reached readily palpable sizes blood was collected from individual mice and carefully fractionated by centrifugation into cellular compartments, such as red blood cells (RBCs), white blood cells (WBCs, buffy coats) and platelets (PLTs), while platelet poor plasma (PPP) was further separated by ultracentrifugation into the EV pellet and EV-free plasma supernatant (SUP). The DNA was extracted from these respective blood compartments and human oncogene (HRAS or HER2) copy number per ml of mouse blood was assessed using sequence specific droplet digital PCR (ddPCR) protocol (Chennakrishnaiah et al., 2018). Surprisingly, while EV and SUP fractions predictably contained oncogenic DNA, as did PLTs, the content of cancer-related genomic sequences were the highest in the WBC fraction, while RBC were virtually devoid of this signal. The contribution of CTC contamination was ruled out through the use of fluorescently labelled cancer cells. Furthermore, the circulating levels of cancer-specific DNA (csDNA) contained in the WBC fraction were higher than those recovered from the liver, spleen or bone marrow, organs where the uptake of EVs is thought to take place, suggesting that it is the circulating fraction of WBCs that sequesters this oncogenic material (Chennakrishnaiah et al., 2018).

Of note is the fact that in small blood samples (up to 100 ul) collected serially from mice harboring RAS3 tumors, the amount of HRAS DNA at the baseline was far more robust in WBCs than the signal recovered from the corresponding cell-free serum. Moreover, a surgical removal of the primary tumor led to extinction of the WBC-associated HRAS DNA signal within 2–3 days (estimated half life of these cells), while the signal in serum remained low and changed minimally over time. This suggests that, at least in some settings, the WBC content of csDNA may serve as a far more robust source of biologically meaningful representation of the driver mutation than csDNA contained in cell-free serum or in plasma (Chennakrishnaiah et al., 2018).

To understand which WBC population may have taken a role of the apparent reservoir of csDNA, buffy coat cellular isolates from blood of RAS3 tumor-bearing mice were sorted into neutrophils, monocytes and lymphocytes using appropriate markers. Interestingly, the greatest amount of human HRAS DNA was found in neutrophils, and the least in lymphocytes, as measured both per blood volume and per cell. This is understandable as neutrophils (and monocytes) possess a professional phagocytic activity and could play a role in clearing circulating particulate matter containing tumor DNA. Moreover, systemic depletion of neutrophils using anti-Ly6G antibody resulted in a shift of circulating csDNA to the EV and SUP (ctDNA) fractions of blood suggesting that, indeed, these cells control the distribution of tumor-related material in the circulation, possibly by ingesting EV-associated or free extracellular DNA (Chennakrishnaiah et al., 2018).

Interestingly, EVs or particles appear to be required for the uptake of extracellular DNA by leukocytes. This is because incubation of RAS3 cell-derived EVs or nucleosomes with myeloid HL-60 cells in culture resulted in the internalization and retention of tumor DNA in these cells for several days, while soluble DNA purified from EVs failed to penetrate into recipient cells (Chennakrishnaiah et al., 2018). Thus, interactions of EVs with circulating professional phagocytes may lead to the accumulation of EV-related DNA in these cells, which therefore may serve as a unique reservoir of cancer specific biomarkers. This experimental approach termed *leukobiopsy* still remains to be tested in diverse experimental models and in clinical settings to assess its possible diagnostic utility.

There are also several expected limitations that may be associated with this particular prospective diagnostic approach. First, the content of germline nuclear DNA may present dilution challenges with respect to detection of small amounts of cancer-related sequences, especially those without unique mutations. Second, the numbers of leukocytes and their phagocytic activities may vary as a function of chemotherapy, infection, inflammation or myelosuppression (in a similar manner as experimental treatment with anti-Ly6G antibody), all of which could affect the ability of these cells to accumulate and retain cancer-related material. Indeed, different forms of biological regulation are likely a relevant consideration for all liquid biopsy platforms.

## Biological Regulators of Liquid Biopsy Signals

While liquid biopsy is often regarded as a passive manifestation in biofluids of the remotely located tumor mass, several poorly understood processes are likely to control the levels of circulating analytes and their carriers, be it CTCs, EVs or ctDNA. The aforementioned example of experimental leukobiopsy exemplifies at least two levels of such a regulation. First, the uptake of EVs and nucleosomes by leukocytes reduces the levels of cell-free mutant DNA in plasma and shifts it to another blood compartment (WBCs) that is not routinely analysed in this setting. Second, as mentioned, neutrophil depletion dramatically increases the EV and ctDNA content of the mutant HRAS signal in blood (Chennakrishnaiah et al., 2018). Since numbers, compositions and states of myeloid cells in blood are regulated by several cancer associated processes, such as inflammation, secondary infections, immunomodulation, or myelosuppression, including the effects of cytotoxic therapy and radiation, it could be argued that the performance of ctDNA or EV-based liquid biopsy assays may be affected by these conditions.

Similar considerations may apply to tumor-educated platelets as a reservoir of cancer-related macromolecules (e.g. RNA)(In ‘t Veld and Wurdinger, 2019). For example, cancer-associated thrombosis (CAT) is a condition that affects variable numbers of patients with the severity that largely depends on cancer site (Wun and White, 2009), type (Hisada and Mackman, 2017), and molecular subtype (Magnus et al., 2013; Unruh et al., 2016). However, the overall prevalence of CAT is very high as autopsy data estimate it to occur in approximately 50% of cases (Timp et al., 2013). CAT involves either an increase (Haemmerle et al., 2018), or consumptive reduction of circulating platelets (Riedl et al., 2017). The latter is often the case in glioblastoma due to the expression of platelet activating surface glycoprotein, podoplanin, on the surface of cancer cells (Riedl et al., 2017). Interestingly, platelets ingest glioblastoma EVs containing oncogenic transcript for EGFRvIII and carry this signature into the circulation (Nilsson et al., 2011). However, certain subtypes of glioblastoma are spared form CAT, due to protective effects associated with the expression of specific transforming mutations, such as those of isocitrate dehydrogenase (IDH1), a phenotype that correlates with reduced expression of tissue factor, podoplanin and other genes (Unruh et al., 2016; Tawil et al., 2019) and with normal platelet counts (Unruh et al., 2016). It is presently unknown, but remains of great interest whether these events affect the levels of blood-borne cancer biomarkers associated with platelets, EVs, or cell-free nucleic acids.

Chemotherapy and radiation could potentially exert complex influences on liquid biopsy analytes. It is possible that in some instances the amounts of molecularly informative cfDNA or DNA associated with EVs could be increased post-treatment due to cell death processes occurring at the tumor site (Swystun et al., 2011). On the other hand, chemotherapy and radiation often trigger myelosuppression and reduced WBC and platelet counts in the circulation. It is possible, but remains to be thoroughly investigated, that these events may shift the content of circulating cancer DNA from leukocytes or plasma and affect assay sensitivity (Ritch and Wyatt, 2018). Nonetheless, the relationship between the effects of therapeutic interventions and the performance of liquid biopsy platforms requires further study and possibly preanalytical adjustments (e.g. timing of sample collection).

Not all cancer cells with comparable biology release oncogenic proteins and nucleic acids into the circulation. For example, in leukemic cells driven by oncogenic PML-RARa this fusion product triggers profound changes in the molecular repertoire of EVs released into the culture media, but such EVs do not contain measurable amounts of the PML-RARA oncoprotein and neither do they transfer this signal to recipient endothelial cells (Fang et al., 2016). Giant cell tumors of the bone (GCT) release certain amounts of oncogenic DNA with mutant oncohistone sequences (H3.3*^G34W^*), but the levels of this material differ between cell lines and, at least in some cases, sequence specific amplification of DNA contained in EVs is dramatically less efficient than in the case of equivalent amounts of cellular DNA suggesting EV-related biochemical changes or fragmentation (Aprikian – unpublished). Certain cancer cells harboring oncogenic RAS exhibit high level of genetic instability and produce ample cytoplasmic DNA (Dou et al., 2015), which is associated with emission of genomic DNA into the EV fraction of conditioned media (Lee et al., 2014) and into blood of tumor bearing mice (Chennakrishnaiah et al., 2018). This process is likely driven by compromised integrity of the nuclear envelope, instability of the cellular genome, onset of autophagy and other processes (Dou et al., 2015) (Tsering – unpublished). Their regulation might therefore change the emission and detection of extracellular DNA. Tumors driven by other oncogenes may produce lower amounts of EV-associated DNA and the levels of this signal in blood of tumor-bearing mice and in cancer patients may also exhibit considerable variability, impacting the sensitivity of detection and the robustness of the respective liquid biopsy tests.

It is also of note that the choice of biofluids may affect the performance of liquid biopsy assays. For example, while in glioblastoma the detection of tumor-specific mutations is possible in both peripheral blood and cerebrospinal fluid (Al-Nedawi et al., 2008; Skog et al., 2008; Graner et al., 2009; Figueroa et al., 2017), the latter represents the liquid space more proximal to cancer cells, rendering signal detection more robust (Zachariah et al., 2018; Seoane et al., 2019). Thus, a better understanding of biological processes and regulatory mechanisms that control the release of liquid biopsy analytes may hold the key to a more rational use of biofluid sources, molecular signal recovery methods and detection techniques for specific cancers and medical purposes.

## Biological Effects of Liquid Biopsy Analytes

It is increasingly clear that liquid biopsy analytes possess important biological activities, which may add meaning and complexity to their detection. In this regard the emerging biological effects of traditional cancer biomarkers, such as PSA (Niu et al., 2008), or CEA (Bramswig et al., 2013) have attracted recent attention as regulators of cellular growth and angiogenesis. While the contribution of CTCs to metastasis is implicit, their interactions with plasma, platelets and other cells in the circulation may result in additional biological perturbations of significance, for instance in the context of systemic CAT and thrombotic events in cancer patients (Beinse et al., 2017). Similarly, extracellular DNA and chromatin released from cancer cells may induce thrombosis (Swystun et al., 2011) and interfere with the function of leukocytes acting as damage recognition molecular patterns (Swystun and Liaw, 2016).

In some of these instances the oncogenic activity of liquid biopsy-associated macromolecules and their carriers (EVs/EPs) may play a role in biological events. For example, oncogenic EGFR released by cancer cells as cargo of EVs detectable in blood (Montermini et al., 2015) may be taken up by endothelial cells and reprogram their biological responses, including activation of the VEGF pathway and angiogenesis (Al-Nedawi et al., 2009). Detection of RAS mutations in circulating blood of cancer patients remains among the most attractive examples of liquid biopsy developments reported to date (Diehl et al., 2008; Bardelli and Pantel, 2017) with several recent promising follow up studies (Cohen et al., 2018). In many of these instances mutant sequences are found in association with circulating EVs (Thakur et al., 2014). However, in the aforementioned study it was found that while oncogenic RAS drove a release of genomic DNA, as well as mutant RNA and altered protein repertoire of cancer cell-related EVs, these EVs were not only informative as to the existence of oncogenic mutation but also highly bioactive (Lee et al., 2014; Lee et al., 2016). Indeed, the uptake of EVs from RAS-driven cells, but not EVs from their isogenic, non-transformed counterparts by cultured leukocytes, resulted in a dramatic change in phenotype, marked by an increase in procoagulant activity associated with tissue factor and elevated release of interleukin 8 (Chennakrishnaiah et al., 2018). These examples merely signal a much broader question of biological activities associated with liquid biopsy analytes and their carriers including extracellular DNA, RNA and proteins (Siravegna et al., 2017), a question that still requires more extensive studies.

## Conclusions and Future Prospects

It could be argued that a biomarker of a pathological process, such as cancer, would ideally be the molecular driver, or an indispensable and unique attribute of it. Oncogenic mutations would meet these criteria if not for dynamic evolution, molecular complexity and cellular heterogeneity of cancer cell populations, which often also depend on exogenous triggers to manifest their disease-causing potential (Ghajar et al., 2013; Magnus et al., 2014; Martincorena et al., 2015). Still, detection of unique molecular changes occurring in the cancer cell genome and epigenome in real time could carry enormous value in developing more adaptive, personalized and ultimately more effective care for cancer patients.

Cancer cells exteriorize these unique signatures though a multitude of regulated processes ranging from the shedding of CTCs, apoptotic bodies, vesiculation and secretory mechanisms, resulting in the influx of analytes, such as cfDNA and other into remote biofluid compartments (Siravegna et al., 2017). In this article, we argued that the release and biological turnover of this material are not necessarily “unspecific”, steady or passive, but instead multiple regulatory steps may perturb the levels, timing and tumor representation in different liquid biopsy settings (**Figure 2**). These regulatory influences may affect their choice and performance of liquid biopsies and require optimization and/or use of multiple approaches simultaneously (e.g. CTCs and EVs). In this regard, we propose that the sequestration of mutant macromolecules by circulating phagocytes may offer a hitherto unappreciated diagnostic opportunity (leukobiopsy), which while presently experimental, is worthy of further exploration.

**Figure 2:** Regulatory points in extracellular trafficking of oncogenic sequences in cancer (a hypothesis). Genomic DNA and mutant nucleic acids exit cancer cells either through secretory mechanisms, vesiculation or cell death. This material circulates in blood and biofluids as either particles (e.g. nucleosomes) or extracellular vesicles (EVs) and both may be ingested by platelets or white blood cells (WBCs). These cells may therefore act as reservoirs and regulatory mechanisms to control the levels of cancer-related nucleic acids. In addition, processes that influence the state and function of blood cells may influence their storage capacity for cancer-related material and possibly the circulating levels of liquid biopsy analytes (see text for details).

Future efforts will be required to determine whether experimental promise of leukobiopsy will be borne out in the clinical reality and whether there may be advantages (beyond technical) to apply specific liquid biopsy platforms to specific different cancer contexts.

## Author Contributions

SC, JR, SA, and TT wrote the manuscript and contributed ideas.

## Funding

This work was supported by the operating grants from Canadian Institutes for Health Research (CIHR Foundation grant FDN143322) to JR, who is also a recipient of the Jack Cole Chair in Pediatric Hematology/Oncology. Infrastructure funds were provided by the Fonds de Recherche en Santé du Quebec (FRSQ).

## Conflict of Interest

SC and JR filed a patent application for diagnostic use of leukocytes as carriers of cancer-causing mutations.

The remaining authors declare that the research was conducted in the absence of any commercial or financial relationships that could be construed as a potential conflict of interest.
